The article "Etiology of Emergency Visit and In-Hospital Outcomes of Patients with COPD" was published in 2022. Journal: Emerg Med Int.

# Etiology of Emergency Visit and In-Hospital Outcomes of Patients with COPD

**DOI:** 10.1155/2022/8247133

**Published:** 2022-08-29

**Authors:** Xueyang Zhang, Qingtao Zhou, Shengfeng Wang, Qingbian Ma, Yongchang Sun

**Affiliations:** ^1^Department of Respiratory and Critical Care Medicine, Peking University Third Hospital, Beijing, China; ^2^Center for Clinical Epidemiology, Peking University Third Hospital, Beijing, China; ^3^Emergency Department, Peking University Third Hospital, Beijing, China

## Abstract

**Backgrounds:**

Patients with COPD often visit the emergency department (ED) due to exacerbation of respiratory symptoms (dyspnea, cough, and sputum production). Because manifestations of acute exacerbation of COPD (AECOPD) are nonspecific, differential diagnosis is critical in this acute setting. The causes for emergency visiting and the in-hospital outcomes are varied in patients with COPD. This study aimed to investigate the distributions of etiologies and the in-hospital outcomes of patients with COPD who presented to the ED because of exacerbation of respiratory symptoms.

**Methods:**

This was a retrospective study on COPD patients who had visited the ED and been hospitalized in a tertiary hospital because of worsening respiratory symptoms including cough, sputum production, and dyspnea from January 2017 to April 2020. Demographics, clinical manifestations, and laboratory studies in the ED were collected as the baseline data. The primary diagnosis at discharge or death was recorded. The hospitalization settings (general wards and ICU), the in-hospital outcomes, and associated factors were analyzed.

**Results:**

During the study period, 392 patients with COPD (male 302 (77.0%)), with a median age of 78 years, visited the ED and hospitalized in this hospital. The first 3 causes for emergency visit were AECOPD (*n* = 314, 80.1%), acute coronary artery syndrome with or without congestive heart failure (*n* = 24, 6.1%), and pulmonary embolism (*n* = 13, 3.3%). For patients with AECOPD (*n* = 314), 51.6% (*n* = 162) was admitted to ICU, and 6.4% (*n* = 20) died. Multivariate logistic analysis showed that age, atrial fibrillation, NT-pro BNP ≥300 pg/ml, and blood pH <7.3 were independent risk factors for ICU admission. Age, comorbid malignancy, NT-pro BNP ≥1800 pg/ml, and pneumonia on CT scan were independent risk factors for hospital mortality in patients with AECOPD.

**Conclusion:**

In COPD patients visiting the ED because of worsening respiratory symptoms, nearly 20% were due to non-AECOPD causes. For those with AECOPD, age, atrial fibrillation, NT-pro BNP ≥300 pg/ml, and blood pH <7.3 were independent risk factors for ICU admission, while advanced age, underlying malignancy, elevated NT-pro BNP, and pneumonia on CT scan were risk factors for hospital mortality.

## 1. Introduction

Chronic obstructive pulmonary disease (COPD) is a globally prevalent disease [1]. In China, the prevalence of spirometry-diagnosed COPD in adults ≥20 years old was 8.6% in a population-based study [2]. Acute exacerbation, defined as worsening of respiratory symptoms needing change of usual care, is an important event in the natural course of the disease [3]. AECOPD can be classified as mild, moderate, and severe, and severe exacerbation often needs emergency visit and/or hospitalization [4]. However, the diagnosis of AECOPD is based solely on clinical manifestations, which are nonspecific, and therefore differential diagnosis is critical for patients presenting to the emergency department (ED). The hallmark symptom of AECOPD is aggravated dyspnea, which is also a manifestation of other critical diseases, including pulmonary and extra-pulmonary diseases, such as heart failure (HF), pulmonary embolism (PE), cardiac infarction, and pneumothorax. A large observational study in Europe and the Asian-Pacific region for patients presenting to EDs with dyspnea as the main complaint showed that the most common causes were lower respiratory tract infection, HF, AECOPD, and asthma [5]. However, the causes for ED visiting in COPD patients with exacerbated respiratory symptoms (dyspnea, cough, and/or sputum) are rarely studied, though the data are important for differential diagnosis and management in this acute setting. Therefore, we conducted a single-center retrospective cohort study on the causes and outcomes of COPD patients presenting to our ED and hospitalized for exacerbation of respiratory symptoms.

## 2. Patients and Methods

### 2.1. Study Subjects

This was a single-center, retrospective observational study performed in Peking University Third Hospital. Patients with COPD presenting to the ED and hospitalized from January 2017 to April 2020 were consecutively enrolled. The inclusion criteria were (1) age ≥40 years; (2) diagnosis of COPD verified by medical records; (3) presenting with exacerbated respiratory symptoms including dyspnea, cough, and/or sputum production; and (4) hospitalized within 72 h after ED evaluation and management. Patients who died at the ED were excluded.

### 2.2. Data Collection

All hospitalized patients with a diagnosis of COPD were retrieved and their medical records were reviewed, and if they had any ED visit during the study period, they were enrolled in the study. For patients with repeated visits, only the first visit was included for analysis. Baseline data and diagnostic studies at the ED and during hospitalization were collected, including demographics, comorbidities, laboratory tests, chest CT, and echocardiography. The symptoms (cough, sputum production, and dyspnea) were derived from the emergency medical records. Only laboratory results from the first ED visit were included in this study. Based on the emergency diagnosis and the discharge diagnosis, we ascertained the etiology for ED visiting. For patients with AECOPD, underlying diseases were recorded as comorbidities, which served as variates in the analysis. The outcomes were admission to the ward or ICU, length of stay, and survival.

### 2.3. Chest  CT Review

Chest CT scans performed within 72 h after presentation to the ED were collected and analyzed. A radiologist and a pulmonary physician reviewed the CT scans. Signs consistent with pneumonia were identified [6, 7].

### 2.4. Statistical Analysis

Statistical analysis was performed using Stata 16.0 software. Comparison between categorical variables was made using the chi-square test. The independent-samples *t*-test (for normal distribution parameters) and Mann–Whitney *U*-test (for abnormal distribution parameters) were adopted for comparisons of continuous data between two groups. Poisson regression and logistic regression were used to analyze the risk factors for ICU admission and in-hospital mortality for patients with AECOPD. *P* values <0.05 were considered as statistically significant.

## 3. Results

### 3.1. Demographics and Baseline Data

From January 2017 to April 2020, 392 eligible COPD patients, with a median age of 78 years, presented to our ED with the main complaint of worsening respiratory symptoms including cough, sputum production, and dyspnea. The demographics and the baseline data are presented in Table 1.

Male patients (*n* = 302) accounted for 77.0% of the population, and 318 patients (81.1%) were current or former smokers. 25.5% (*n* = 100) of the patients were on family oxygen therapy and/or noninvasive positive pressure ventilation (NIPPV) therapy. The most common comorbidity was hypertension (212, 54.1%), followed by arrhythmia (109, 27.8%) with atrial fibrillation as the most common (71/109, 65.1%), cerebrovascular disease, diabetes, and benign prostatic hyperplasia. Malignancy was present in 53 patients (13.5%), in which 29 patients had lung cancer (the most common). Totally, 319 (81.4%) patients had at least 1 comorbidity and 137 (34.9%) had 3 or more comorbidities. More than half of our patients were using LAMA, ICS, or ICS/LABA.

### 3.2. Distribution of Etiologies for ED Presentation

The primary diagnosis of the causes for ED visiting of the COPD patients complaining of exacerbated respiratory symptoms are outlined in Figure 1 and Figure 2. Most of the patients (*n* = 314, 80.1%) presented to the ED and then hospitalized because of AECOPD. For patients with consistent manifestations and infiltrates on chest CT, we classified them as those with pneumonic AECOPD [6, 7] and hence included in the AECOPD group. It is notable that in our cohort, non-AECOPD accounted for 19.9% of the primary causes for ED presentation, including acute coronary syndrome and/or HF, PE, and pneumothorax.

### 3.3. In-Hospital Outcomes of the Non-AECOPD Patients

Of the 78 patients (19.9%) with non-AECOPD causes for ED visiting, 24 (24/78, 30.8%) were due to acute coronary syndrome and/or HF (8 with reduced ejection fraction), and 2 cases died in hospital. Thirteen patients (13/78, 16.7%) were found to suffer from PE by computed tomography pulmonary angiogram (CTPA) and/or ventilation-perfusion scan. Ten patients (10/78, 12.8%) had pneumothorax, in which 1 was caused by lung puncture for diagnosis of lung lesions and 1 patient died. Eight patients were found to have lung cancer (8/78, 10.3%), among whom two had pleural effusion and 1 had obstructive pneumonia. Six patients (6/78, 7.7%) were confirmed to have fungal pulmonary infection, and 1 died. Other causes and the in-hospital outcomes are shown in Table 2.

### 3.4. In-Hospital Outcomes and Associated Risk Factors of the Patients with AECOPD

#### 3.4.1. Demographics and Baseline Data of the Patients with AECOPD

Among the 314 patients presenting to the ED and were hospitalized for AECOPD, there were 242 males (77.1%, 242/314), with a median age of 78 years; 54 (17.2%, 54/314) aging <65 years, 133 (42.4%, 133/314) aging 65–80 years, and 127 (40.4%, 127/314) aging >80 years. A quarter of them (*n* = 78) were receiving long-term oxygen therapy or NIPPV. As in the whole population, hypertension, arrhythmia, and cerebrovascular disease (CVD) were the 3 most common comorbidities (see Table 3).

In the ED evaluation, higher WBC (>10 × 10^9^/L) was found in 148 patients (48.5%, 148/305), anemia (Hb <120 g/dl) in 20.7% (63/305), and higher PCT (>0.25 *μ*g/ml) in 41.6% patients (79/190). Eighty-six patients (32.1%, 86/268) had a NT-pro BNP level ≥1800 pg/ml, while NT-pro BNP <300 pg/ml was present in 81 patients (30.2%, 81/268). Blood gas analysis showed pH <7.35 in 26.7% patients (75/281), and 43 patients had pH <7.3 (43/281, 15.3%). 45.2% patients had PaCO_2_ greater than 50 mmHg (127/281). We found that a total of 70 patients (70/281, 24.9%) had pH <7.35 with PaCO_2_ >50 mmHg. 249 patients had chest CT taken within 72 h after presentation to the ED, and the results revealed infiltrates consistent with clinical pneumonia in 95 (38.2%, 95/249) (Table 3).

#### 3.4.2. In-Hospital Outcomes of the AECOPD Patients

Of the AECOPD patients presenting to the ED, more than half (51.6%, 162/314) were admitted to ICU, and others (152, 48.4%) were admitted to the general ward. Among patients in the ward, 5 died; and among those in ICU, 15 died, resulting in a total in-hospital mortality of 6.4% (20/314). The median length of stay in ICU was 15 days (interquartile range, IQR 11–22), and the length of stay in hospital of all the patients was 13 days (IQR 10–19).

#### 3.4.3. Risk Factors for ICU Admission and In-Hospital Mortality in AECOPD Patients Presenting to the ED

Comparison between patients admitted to ICU and the general ward is shown in Table 3. Patients admitted to the ICU were older and had higher levels of D-dimer, PCT, and NT-pro BNP, and more patients had ≥2 comorbidities, arrhythmia or HF. Because the latest heart failure guidelines recommend NT-pro BNP <300 pg/ml as a threshold to exclude heart failure in emergency situations [8], we used this cut-off value for analysis. The results showed that age (odds ratio (OR) 1.04, 95% confidence interval (CI) 1.005–1.069, *P* value 0.021), atrial fibrillation (OR 2.99, 95% CI 1.16–7.71, *P* value 0.023), NT-pro BNP ≥300 pg/ml (OR 2.58, 95% CI 1.38–4.80, *P* value 0.003), and pH <7.3 (OR 8.73, 95% CI 2.35–32.4, *P* value 0.001) were independent risk factors for ICU admission.

Comparison between survivors and nonsurvivors in hospital is shown in Table 3. Malignancy, HF, and arrhythmia were significantly different between the two groups. Because the cut-off value of NT-pro BNP for the diagnosis of acute heart failure was age-dependent, i.e., ≥ 450 pg/ml (<50 years old), ≥900 pg/ml (50∼75 years old), and ≥1800 pg/ml (>75 years old), respectively, for different age groups [9], we used NT-pro BNP ≥1800 pg/ml for analysis as the median age of our cohort was older than 75 years. The results showed that age (incidence rate ratio (IRR) 1.08, 95% CI 1.02–1.16, *P* value 0.013), malignancy (IRR 6.0, 95% CI 2.14–16.87, *P* value 0.001), NT-pro BNP ≥1800 pg/ml (IRR 6.09, 95% CI 2.2–16.88, *P* value 0.001), and pneumonia on CT scan (IRR 3.52, 95% CI 1.40–8.81, *P* value 0.007) were independent risk factors for hospital mortality.

## 4. Discussion

AECOPD is defined as an acute worsening of respiratory symptoms resulting in additional therapy. As comorbidities that may worsen respiratory symptoms are common in COPD patients, clinical assessments to rule out alternative diagnoses should be performed before confirmation of a COPD exacerbation [10]. In clinical practice, because patients with COPD often visit the ED due to exacerbation of respiratory symptoms, differential diagnosis is critical in this acute setting. However, detailed, practical studies of the causes for ED visiting in the COPD population are scarce. Here, we described the distributions of etiologies and the in-hospital outcomes of patients with COPD who presented to the ED because of exacerbation of respiratory symptoms. We found that the top five causes for ED visiting in our cohort were AECOPD, acute coronary syndrome and/or heart failure, PE, pneumothorax, and lung cancer, confirmed after careful examinations in the ED and after hospitalization. We also found that advanced age, malignancy, atrial fibrillation, elevated NT-pro BNP, pH <7.3, and pneumonia on CT scans increased the risk of ICU admission and/or in-hospital mortality in patients with AECOPD.

A large population-based study in Canada showed that, for the 27,705 admissions with a diagnosis of COPD at the EDs, the primary diagnoses at discharge were mostly related to COPD per se (*n* = 20, 848, 75.2%), followed by pulmonary infections (*n* = 2916, 10.5%). Cardiac conditions including heart failure, ischemic heart disease, or chest pain represented 8.3% of the admissions (*n* = 2311, 8.3%). Other serious conditions complicating COPD (for example, pneumothorax, PE, or stroke) were reported infrequently (*n* = 129, 0.5%) [11]. However, this study was based on provincial administrative databases, which lacked detailed clinical information at the EDs. In a recent study on COPD patients admitted to the hospital due to acute worsening of respiratory symptoms, PE was detected in 5.9% of patients using a predefined diagnostic algorithm [12]. The pooled prevalence of PE in “unexplained” AECOPD was 16.1% (95% CI, 8.3%–25.8%) in a total of 880 patients [13].

Current guidelines recommend that patients suspected with AECOPD should be differentiated from diagnosis of pneumonia, pneumothorax, PE, cardiac events, and arrhythmia [10]. As COPD patients with exacerbated respiratory symptoms often present to the EDs, our results provided practical data for emergency physicians to differentiate AECOPD from other causes and to start proper treatment in time at this acute setting.

Smoking and aging are common risk factors for COPD and other chronic diseases, which are associated with multiple comorbidities in COPD [14]. The prevalence of HF in COPD patients ranges from 7.1% to 31.3%, and the prevalence of coronary heart diseases (including myocardial infarction, angina, and ischemic heart disease) ranges from 4.7% to 60% [15]. Cardiac complications were highly associated with an increased risk of death [16] in COPD patients. In this study, our findings were consistent with others in terms of the risk factors for ICU admission and in-hospital mortality in patients with AECOPD, including older age [17], cardiovascular complications [18] (arrhythmia, HF), malignancy [16], pneumonia [19–21], anemia [22], and high levels of NT-pro BNP [23].

BNP has moderate accuracy in detecting HF in the EDs [24], but interestingly, NT-pro BNP was a strong and independent predictor of in-hospital mortality in AECOPD patients [25]. Buchan et al. found that elevated BNP or NT-pro BNP levels in AECOPD were associated with increased mortality from cardiovascular diseases [26]. An earlier study showed that AECOPD was definitely associated with acute left-heart dysfunction in 31.1% and possibly with left ventricular dysfunction in 13.5% of the patients [27]. Furthermore, COPD is associated with a high incidence of pulmonary hypertension, which is linked with exercise limitation and a worse prognosis [27]. In AECOPD patients without underlying left ventricular dysfunction, log-transformed NT-pro BNP levels were positively associated with echocardiographically estimated right ventricular systolic pressure [28]. It should be noted that the NT-pro BNP cut-off values for assessing ICU admission and in-hospital mortality were different in our study because the diagnostic threshold of NT-pro BNP was varied. A level <300 pg/ml is often used to rule out HF [8]. When it comes to assessing in-hospital mortality, the diagnosis of HF is more important. Therefore, we used NT-pro BNP ≥1800 pg/ml for analysis of in-hospital mortality, as the median age of our cohort was older than 75 years. In addition, in this study, we used two regression models for analysis of the risk factors because the number of patients who died in hospital was relatively small. Poisson regression and logistic regression were used at the same time to make the regression result more robust, and the two regression results were similar.

Our study had several limitations. As a retrospective study, some examination results and lab data were not available for all our patients. In this hospital, patients requiring noninvasive or invasive mechanical ventilation were all admitted to ICU, and therefore the ICU admission rate was high. As a single-center study, the sample size was relatively small, and the results may not be applicable to other ED practice.

## 5. Conclusion

Our study found that, for COPD patients who presented to the EDs because of exacerbated respiratory symptoms, non-AECOPD causes accounted for about 20%, most commonly acute coronary syndrome and/or heart failure, and PE. For patients with AECOPD, age, atrial fibrillation, NT-pro BNP ≥300 pg/ml, and blood pH <7.3 were independent risk factors for ICU admission, while advanced age, underlying malignancy, NT-pro BNP ≥1800 pg/ml, and pneumonia on CT scan increased the risk of in-hospital mortality.

## Figures and Tables

**Figure 1:** The discharge diagnosis of the patients. ED: emergency department; AECOPD: acute exacerbation of chronic obstructive pulmonary disease; ICU: intensive care unit; RA: rheumatoid arthritis.

**Figure 2:** Distribution of the primary causes for ED presentation of the 392 COPD patients.

**Table 1:** Demographics, baseline, and comorbidity data of the patients.

	Patients (*N* = 392)
Age, (median, range)	78 (70–84)

Male, *n* (%)	302 (77.0)

Current and former smokers, *n* (%)	318 (81.1)

LTOT, *n* (%)	100 (25.5)

*Medications for COPD*	
ICS + LABA + LAMA	94 (24.0)
Theophylline + ICS + LABA + LAMA	70 (17.9)
LAMA	38 (9.7)
ICS + LABA	30 (7.7)
Theophylline + ICS + LABA	18 (4.6)
Theophylline	11 (2.8)
Theophylline + LAMA	5 (1.3)

*Comorbidity, n (%)*	
No comorbidity	73 (18.6)
1 comorbidity	82 (20.9)
2 comorbidities	100 (25.5)
≥3 comorbidities	137 (34.9)
Hypertension	212 (54.1)
Arrhythmia	109 (27.8)
Coronary artery disease	78 (19.9)
Old MI	19 (4.8)
After PCI	22 (5.6)
Cerebrovascular disease	78 (19.9)
Diabetes mellitus	77 (19.6)
BPH	67 (17.1)
Malignancy	53 (13.5)
Congestive heart failure	39 (9.9)
Asthma	35 (8.9)
CRF	26 (6.6)
Hyperlipidemia	25 (6.4)
GERD	19 (4.8)
Gastric/duodenal ulcers	16 (4.1)

LTOT: long-term oxygen therapy; PCI: percutaneous coronary intervention; BPH: benign prostatic hyperplasia; GERD: gastroesophageal reflux disease; MI: myocardial infarction; CRF: chronic renal failure; LAMA: long-acting muscarinic antagonist; LABA: long-acting *β*2-agonist; ICS: inhaled corticosteroid; OCS: oral corticosteroid; Ca2 + RA: calcium receptor antagonist; ACE-I: angiotensin-converting enzyme inhibitor; ARB: angiotensin receptor blocker.

**Table 2:** Non-AECOPD causes for ED presentation and in-hospital outcomes of the 78 COPD patients.

Diagnosis	No. (%) (*N* = 78)	Discharged (%)	Died (%)
Acute coronary syndrome and/or heart failure	24 (30.8)	22 (28.2)	2 (2.6)
Pulmonary embolism	13 (16.7)	13 (16.7)	0 (0)
Pneumothorax	10 (12.8)	9 (11.5)	1 (1.3)
Lung cancer	8 (10.3)	8 (10.3)	0 (0)
Pulmonary fungal infection	6 (7.7)	5 (6.4)	1 (1.3)
Tuberculosis/tuberculous pleurisy	5 (6.4)	4 (5.1)	1 (1.3)
Lung abscess	3 (3.8)	3 (3.8)	0 (0)
Haemoptysis cause undetermined	2 (2.6)	0 (0)	2 (2.6)
Septic shock	2 (2.6)	1 (1.3)	1 (1.3)
Organizing pneumonia	2 (2.6)	2 (2.6)	0 (0)
Rheumatoid arthritis-associated lung disease	1 (1.3)	1 (1.3)	0 (0)
Granulomatosis with polyangiitis	1 (1.3)	1 (1.3)	0 (0)
Tracheal stenosis	1 (1.3)	1 (1.3)	0 (0)

**Table 3:** Comparisons between patients with AECOPD admitted to ICU or general wards, survivors, or nonsurvivors.

Variable	*n*	AECOPD (314)	ICU (162)	General wards (152)	*P* values	Survival (294)	In-hospital mortality (20)	*P* values
Male, *n* (%)	314	242 (77.1)	114 (70.4)	128 (84.2)	0.004	225 (76.5)	17 (85.0)	0.384
Age (median, range)	314	78 (69–84)	80 (71–86)	77 (66–82)	<0.001	78 (69–83)	84.5 (73–90.5)	0.012
Age <65 yr		54 (17.2)	17 (10.5)	37 (24.3)	Reference	52 (17.7)	2 (10.0)	Reference
65 yr ≤age <80 yr		133 (42.4)	65 (40.1)	68 (44.7)	0.032	126 (42.9)	7 (35.0)	0.655
Age ≥80 yr		127 (40.4)	80 (49.4)	47 (30.9)	<0.001	116 (39.5)	11 (55.0)	0.259
Current/former smoker	314	253 (80.6)	126 (77.8)	127 (83.6)	0.196	238 (81)	15 (75.0)	0.515
LTOT	314	78 (24.8)	50 (30.9)	28 (11.8)	0.011	75 (25.5)	3 (15.0)	0.293
Comorbidity	314							
No comorbidity		63 (20.1)	24 (14.8)	39 (25.7)	Reference	63 (21.4)	0 (0)	
1 comorbidity		66 (21.0)	30 (18.5)	36 (23.7)	0.398	64 (22.4)	2 (10.0)	Reference
2 comorbidities		84 (26.8)	49 (30.2)	35 (23.0)	0.016	74 (25.2)	10 (50.0)	0.008
≥3 comorbidities		101 (32.2)	59 (36.4)	42 (27.6)	0.012	93 (31.6)	8 (40.0)	0.037
Hypertension		163 (51.4)	90 (55.6)	73 (48.0)	0.182	152 (51.7)	11 (55.0)	0.775
Arrhythmia		78 (24.8)	53 (32.7)	25 (16.4)	0.001	68 (23.1)	10 (50.0)	0.007
Coronary artery disease		65 (20.7)	35 (21.6)	30 (19.7)	0.683	61 (20.7)	4 (20.0)	0.936
Old MI		15 (4.8)	9 (5.5)	6 (3.9)	0.504	15 (5.1)	0 (0)	0.301
After PCI		17 (5.4)	8 (4.9)	9 (5.9)	0.701	16 (5.4)	1 (5.0)	0.933
Cerebrovascular disease		61 (19.4)	33 (20.4)	28 (18.4)	0.663	59 (20.1)	2 (10.0)	0.271
Diabetes mellitus		55 (17.5)	34 (21.0)	21 (13.8)	0.095	53 (18)	2 (10.0)	0.361
BPH		57 (18.2)	26 (16.0)	31 (20.4)	0.318	54 (18.4)	3 (15.0)	0.705
Malignancy		35 (11.1)	20 (12.3)	15 (9.9)	0.486	26 (8.8)	9 (45.0)	<0.001
Congestive heart failure		32 (10.2)	23 (14.2)	9 (6.0)	0.015	26 (8.8)	6 (30.0)	0.002
Asthma		31 (9.9)	11 (6.8)	20 (13.2)	0.059	31 (10.5)	0 (0.0)	0.126
CRF		17 (5.4)	12 (7.4)	5 (3.3)	0.107	16 (5.4)	1 (5.0)	0.933
Hyperlipidemia		23 (7.3)	12 (7.4)	11 (7.2)	0.954	23 (7.8)	0 (0.0)	0.194
GERD		16 (5.1)	5 (3.1)	11 (7.2)	0.095	16 (5.4)	0 (0.0)	0.284
Gastric/duodenal ulcers		8 (2.5)	6 (3.7)	2 (1.3)	0.180	7 (2.4)	1 (5.0)	0.472
Laboratory studies	314							
Hemoglobin (g/L)	305	137 (123–151)	134 (120–151)	140 (125–150)	0.150	138 (124–151)	120 (98–139)	0.001
WBC count (×10^9^/L)	305	9.8 (7.3–13.5)	10.2 (7.3–13.5)	9.63 (7.4–13.36)	0.763	9.7 (7.2–13.2)	12.7 (9.1–16.1)	0.028
Neutrophils (×10^9^/L)	305	7.8 (5.1–11.1)	8 (4.9–11.2)	7.4 (5.4–11.0)	0.532	7.5 (5–11)	10.1 (7.4–14.2)	0.030
Lymphocytes (×10^9^/L)	305	0.99 (0.67–1.47)	0.91 (0.59–1.35)	1.07 (0.76–1.62)	0.020	0.99 (6.2–16.8)	1 (0.46–1.36)	0.538
Fibrinogen (mg/dl)	242	4.13 (3.35–4.98)	4.06 (3.28–4.86)	4.32 (3.44–5.48)	0.199	4.08 (3.32–4.98)	4.37 (3.92–5.57)	0.17
D-dimer (*μ*g/ml)	283	0.31 (0.17–0.61)	0.40 (0.20–0.78)	0.24 (0.15–0.44)	<0.001	0.29 (0.17–0.57)	0.71 (0.29–2.29)	0.001
PCT (*n*g/ml)	190	0.183 (0.11–0.76)	0.2 (0.12–1)	0.13 (0.1–0.48)	0.003	0.175 (0.1–0.72)	0.25 (0.15–3.55)	0.144
NT-pro BNP (pg/ml)	268	753.5 (229–2300)	1480 (504–4010)	310 (136–856)	<0.001	735 (202–2060)	4540 (2370–7920)	<0.001
CK-MB (U/liter)	298	14 (9–20)	15 (11–22)	13 (9–18)	0.024	14 (10–20)	14 (8.5–25)	0.789
Arterial blood gas	281							
pH		7.41 (7.34–7.45)	7.36 (7.3–7.43)	7.43 (7.4–7.46)	<0.001	7.41 (7.34–7.45)	7.39 (7.29–7.45)	0.526
PaCO_2_		48 (38–64)	59 (45–75)	40 (35.3–47)	<0.001	48 (38–65)	45 (37–56)	0.280
PaO_2_		57 (42–73)	54 (38–71)	61 (48.5–75.85)	0.001	57 (43–73)	60.5 (39–76)	0.880
Chest CT	249		116	133		234	15	
Pneumonia		95 (38.2)	48 (41.4)	47 (31)	0.803	86 (36.8)	9 (60)	0.138

^*∗*^Data are presented as median (interquartile range) for continuous variables and No. (%) for categorical variables, unless indicated otherwise. LTOT: long-term oxygen therapy; PCI: percutaneous coronary intervention; BPH: benign prostatic hyperplasia; GERD: gastroesophageal reflux disease; CRF: chronic renal failure; MI: myocardial infarction; PCT: procalcitonin; WBC: white blood cell.

## Data Availability

The data sets used and/or analyzed during the current study are available from the corresponding authors on reasonable request.

## Abbreviations

OR: Odds ratios
CI: Confidence intervals
SD: Standard deviation
ED: Emergency department
IQR: Interquartile range
ICU: Intensive care unit
BNP: B-type natriuretic peptide
NT-pro BNP: N-terminal pro-brain natriuretic peptide
IRR: Incidence rate ratio
COPD: Chronic obstructive pulmonary disease
AECOPD: acute exacerbation of COPD
HF: Heart failure
PE: pulmonary embolism
CVD: Cerebrovascular disease
NIPPV: Noninvasive positive pressure ventilation
CT: Computed tomography
CTPA: Computed tomography pulmonary angiogram.
